The article "Analysis of Students' Role Perceptions and their Tendencies in Classroom Education Based on Visual Inspection" was retracted in 2024. Reasons: signs of a paper mill; suspected computer-generated content; unreliable results or conclusions; lack of ethics approval or compliance.

# Analysis of Students' Role Perceptions and their Tendencies in Classroom Education Based on Visual Inspection

**DOI:** 10.1155/2022/3650308

**Published:** 2022-04-14

**Authors:** Lanlan Jiang

**Affiliations:** Institute of Marxism and Research, Jiangxi Police College, Nanchang Jiangxi 330000, China

## Abstract

This paper presents an in-depth study and analysis of students' role perceptions and their tendencies in classroom education using a visual inspection approach. A multi example learning student engagement assessment method based on a one-dimensional convolutional neural network is proposed. Based on the conceptual composition of student engagement, head posture, eye gaze, and eye-opening and closing states and the most used facial movement units are used as visual features. For feature extraction, the proposed view of relative change features, based on the video features extracted from the Open Face toolset, the standard deviation of the distance between adjacent multiple frames relative to the center point of the three visual features is used as the relative change features of the video. This results in the phenomenon that students are highly motivated in the early stage and significantly increase the rate of absenteeism in the later stage. With the development of information technology injecting new vitality into educational innovation, many researchers have introduced computer vision and image processing technology into students' online learning activities, and understand students' current learning situation by analyzing students' learning status. There are relatively few studies in this area in classroom teaching. Considering the low relative position correlation of the features in the examples, the examples are analyzed using a one-dimensional convolutional neural network to obtain the example-level student engagement, and a multi-example pooling layer is used to infer the student engagement in the video from the example-level student engagement. Finally, the experimental method is used to apply the student classroom attention evaluation detection system to actual classroom teaching activities, and the effectiveness and accuracy of the design of the student classroom attention evaluation detection system are investigated in depth through specific applications and example analysis, and the accuracy of the method of this paper is further verified by communicating feedback with teachers and students in the form of interviews.

## 1. Introduction

The rapid popularization of the Internet has given rise to a continuous change in educational resources, and the emergence of various online teaching resources has enabled students to break the constraints of time and space to freely choose the subjects they are interested in for learning, which has greatly enriched their learning styles. However, there are also some problems with online classroom teaching, because of the weak constraint of online teaching, resulting in the phenomenon of students' high motivation in the early stage and significantly higher absence rate in the later stage [1]. Make synchronized classroom videos more fun, interactive, and experiential. For Internet education, it is very necessary to use deep learning computer vision technology to improve the quality of Internet education courses. Therefore, the introduction of intelligent technology to collect students' learning behaviors, analyze students' learning situations, and make comprehensive process evaluation of students, based on the evaluation results, teachers can understand students' learning situation in time and adjust teaching contents and strategies according to the right remedy, which is of great research value to improve students' overall learning quality [2]. The use of a manual recording of teaching videos has great limitations for many recordings, and the recorded video is only a single, boring record of the classroom. Therefore, automation, intelligence, and interactivity of the recording process are of great importance for synchronous classroom recording. The application of an intelligent and automatic recording system can better record the teacher's lecture, students' listening, and students' interaction with the teacher, making the synchronous classroom video more interesting, interactive, and experiential. For Internet education, it is necessary to use computer vision technology of deep learning to improve the quality of Internet education courses.

The article "Analysis of Students' Role Perceptions and their Tendencies in Classroom Education Based on Visual Inspection" was retracted in 2024. Reasons: signs of a paper mill; suspected computer-generated content; unreliable results or conclusions; lack of ethics approval or compliance.

In the classroom teaching process, teachers can understand the current attention of students through the change of their head posture, and determine in time whether students' eyes focused on the blackboard area and whether they are distracted and deserting. For the students, by paying attention to the teacher's head posture, they can understand the teacher's attention direction in time to realize the information interaction between the teacher and the students [3]. In addition, psychological studies have found a correlation between the direction of human head posture and psychological state. The study of students' head posture has become an important research direction to focus on the change of students' learning status, and through the study of students' head posture, we can understand students' learning status and make early decisions to promote students' development. At the same time, it has very important application value and research significance for intelligent modern education theory research.

The article "Analysis of Students' Role Perceptions and their Tendencies in Classroom Education Based on Visual Inspection" was retracted in 2024. Reasons: signs of a paper mill; suspected computer-generated content; unreliable results or conclusions; lack of ethics approval or compliance.

At present, a large part of the online education resources on the Internet platform manually recorded videos of single teachers' lectures, which not only consume human and material resources but also have serious homogenization [4]. With the development of machine learning, computer vision, deep learning, and other technologies as well as hardware devices, we can take different forms of information captured by the camera as an input to the computer, and through a series of algorithms such as deep learning and computer vision, the computer can have the ability to understand the information like a human, to obtain the results we need. In this paper, we use machine learning and deep learning methods to visually detect the lecturer and rising students in the classroom to restore the classroom teaching more realistically, which has a very positive effect and impact on the synchronous classroom on the Internet. The time and space separation of teachers and students is a significant feature of AI online education, which has advantages and disadvantages, bringing us a convenient new type of education, but also creating the problem of difficulty to evaluate the effectiveness of education. We know that the evaluation of classroom teaching effect can be determined by students' status, and in the classroom context, students' concentration on the classroom is the primary requirement for education, so concentration judgment becomes one of the necessary ways to monitor the classroom effect. By judging students' concentration in the video content, we can solve the problem of unmonitored students' status in the classroom, and effectively detect when students do not appear in front of the camera or doze off during the class. Therefore, concentration detection has great research significance for the part of emotional deficiency in the process of online education.

## 2. Related Work

The method based on eyesight tracking mainly uses professional equipment to capture the relationship between eye rotation, pupil change, and blink frequency to determine whether the test subject's sight is focused on a specific area, and if the test subject's sight is focused on the classroom screen can indicate that the test subject's concentration is focused in the classroom [5]. The video and caption layout are used as independent variables based on the MOOC teaching interface to analyze students' attention problems in online education mainly through eye movements. Eye movement recognition combined with expression recognition to count eye blinks and pupil changes to determine the learners' wakefulness, interest, and pleasure levels, and thus evaluate the classroom [6]. The same study analyzes students' eye movements and concentration levels, and they use specialized eye-movement equipment to obtain information. This type of method has good results, but since ordinary camera equipment cannot capture eye and pupil movements, a major feature of this type of method is that it requires professional equipment to obtain students' eye characteristics and track eye rotation to determine the learners' activity level, so it has some reference value in experimental settings and specific scenarios. However, this type of method has some limitations because online education using objects may use different devices [7].

The article "Analysis of Students' Role Perceptions and their Tendencies in Classroom Education Based on Visual Inspection" was retracted in 2024. Reasons: signs of a paper mill; suspected computer-generated content; unreliable results or conclusions; lack of ethics approval or compliance.

It is believed that knowledge is massive and accessible under the Internet model, and such a feature brings convenience while often generating many disturbing factors. Primary and secondary school students, who cannot discriminate, are more likely to be overwhelmed by the vast amount of information and even go astray. Teachers need to become the discriminators of quality knowledge and the guardians of students [8]. At the same time, it has very important application value and research significance for the research of intelligent modern education theory. The role of teachers in the “Internet+” context is diverse. Firstly, teachers are mentors of students, and secondly, they should be lifelong learners, practitioners, and reflectors. In the Internet era, teachers should take on the roles of teaching instructor, student guide, designer, and researcher. Some of these were already in place in the traditional era, but networking has given them new characteristics [9].

The researcher also suggests that a scientific assessment system is a basis for effective teacher management and that teachers should take advantage of the technology of the Internet to conduct a scientific and systematic assessment of the whole process of student learning, and at the same time, teachers should focus on managing the mixed educational information in the Internet+ environment, i.e., screening and analyzing the huge amount of educational information [10]. The Internet is a tool for teachers and students to learn from each other. Teachers and students become a learning community [11]. In any era, teachers must continue to improve their knowledge system. In the new era, the educational environment and educational resources are moving from closed to open, so teachers should use the technical support of the Internet to learn in-depth and lifelong learning. Teachers need to become good users of network technology. In terms of teacher-student interaction, teachers' pay close attention to the psychological state of learning based on the completion of communication and communication with students, avoiding the use of technology that reduces the opportunities for face-to-face communication between teachers and students, and emphasizing the need for teachers to understand students and grasp their emotional trends. The researcher believes that the role of the teacher is not - unchanging and should be given new connotations of the role with the development of the times.

The article "Analysis of Students' Role Perceptions and their Tendencies in Classroom Education Based on Visual Inspection" was retracted in 2024. Reasons: signs of a paper mill; suspected computer-generated content; unreliable results or conclusions; lack of ethics approval or compliance.

## 3. Analysis of Students' Role Perceptions and their Tendencies in the Classroom Education of Visual Detection Methods

### 3.1. Analysis of Visual Detection Tendency Analysis Algorithm

The face detection method based on a priori knowledge is to apply certain face detection rules and methods to accurately describe the features of various faces and their interrelationships. For example, if two facial features of a person exist in a face image at the same time, and in the face, a priori features it is usually assumed that a nose, a mouth, and a set of symmetrical eyes will exist on the face [12]. This detection method has certain problems, it relies on clear machine recognition rules, and the establishment of machine recognition rules is a complex process, if the face detection rules formulated too strictly, it may directly cause the failure of face detection because it cannot pass all the rules; if the face detection rules are vague and too general, some wrong information may be accepted to affect the detection accuracy. Moreover, the external environment factors are diverse, and it is impossible to apply a unified detection rule to describe all face information. Therefore, this research method can only be used for face detection under some simple backgrounds and fixed poses.

Since the face detector was proposed, methods such as integral map, and cascade structure have rapidly become the main tools for face detection. There are certain problems with this detection method. It relies on clear machine identification rules, and the establishment of machine identification rules is a complex process. If the face detection rules are made too strict, they cannot pass the detection of all rules, it may directly cause the failure of face detection; if the face detection rules are vague and too general.

PARCLOS detects the percentage of time in which the eye is closed for a specified unit of time that exceeds a threshold value f as a percentage of the total time. Due to the different settings of the threshold f, its detection models are generally divided into three types: P70 (f =70%), P80 (f =80%), and EM (f =50%), and the only difference is that the three methods differ in the defined area when the eye is closed when conducting experiments, with P70, P80, and EM indicating a closed area of more than 70%, 80%, and 50%, respectively.

The article "Analysis of Students' Role Perceptions and their Tendencies in Classroom Education Based on Visual Inspection" was retracted in 2024. Reasons: signs of a paper mill; suspected computer-generated content; unreliable results or conclusions; lack of ethics approval or compliance.

The distribution of training data weights is first initialized and then these classifiers are trained. If the data are correctly classified by the classifier to be trained during the training process, then the corresponding weights are changed when the dataset is constructed next, and the whole training process is iterated. The data weights are initialized, given a weight of 1/*N* for each sample.

(1) $$\begin{array}{c} D_{1}=\left(w_{11},w_{12},\cdots ,w_{1i},w_{1N}\right),\;i\in N \end{array}$$

In practical applications, a single strong classifier is difficult to obtain in training, but Adaboost can achieve this by combining weak classifiers, which has the advantages of high interference resistance, fast detection, and high accuracy of the strong classifier after iteration [13]. At present, the mainstream Adaboost weak classifiers are decision trees and neural networks, which have the advantages of being able to freely combine various regression classification models, flexible structure, and not easy to overfit.

(2) $$\begin{array}{c} G\left(x\right)=\mathrm{sign}\left(f\left(x^{2}\right)\right) \end{array}$$

The number of features to be computed in an image is very large, and the use of an integral grayscale map can greatly speed up the computation of Hear-like features because it can accurately describe the global information of the face image, thus shortening the workload and time for training the face image detector, and improving the speed of face image detection. The representation of the integrated gray value magnitude of the pixel in the image feature value is shown in Figure 1.

After calculating the weights of Hear-like feature samples, multiple optimal weak classifiers need to be trained to form a strong classifier, and the weaker classifier feature samples are trained, the higher the accuracy of the final strong classifier sample detection results. The first time the classifier is trained, each sample is set to the same weight, and through the training, the wrong sample and the correct sample are set to different weights, and the weight of the wrong sample is increased and the weight of the correct sample is decreased so that the corresponding multiple weak classifiers can be obtained directly after several cycles, and the strong classifier can be obtained by combining these weak classifiers according to the proportion of the relative sample weights. To enhance the accuracy of face detection, it is usually necessary to train multiple strong classifiers and form them into a cascade classifier [14]. P70, P80, and EM represent closed areas exceeding 70%, 80%, and 50%, respectively. By inputting the sample data into the cascade classifier sequentially, face detection is achieved by detecting the tracking recognition of human and non-human faces.

The article "Analysis of Students' Role Perceptions and their Tendencies in Classroom Education Based on Visual Inspection" was retracted in 2024. Reasons: signs of a paper mill; suspected computer-generated content; unreliable results or conclusions; lack of ethics approval or compliance.

For each Hear-like feature, j corresponds to a weak classifier *h*_*i*_(*x*) expressed in the formula as equation (3): where *x* is the window to be detected, *f*_*i*_(*x*) is the feature value, *p*_*i*_is the direction of the inequality, and *ϕ* represents the threshold value.

(3) $$\begin{array}{c} h_{i}\left(x\right)=\left\{\begin{array}{cc} 1, & p_{i}f_{i}\left(x\right)\geq p_{i}\phi \\ 0, & other \end{array}\right. \end{array}$$

The combination formula for the strong classifier is as follows, where *a*_*t*_^2^ is the weight size of the corresponding weak classifier.

(4) $$\begin{array}{c} F\left(x\right)=\mathrm{sign}\left(\overset{T}{\underset{t=1}{\sum }}a_{t}^{2}h_{t}\left(x\right)\right) \end{array}$$

In the image tracking of the window of a face target in the next video frame search image, the parameters of the current video frame search window are reset and initialized using the second-order values of the obtained search window, and the second-order moments of the search window are:

(5) $$\begin{array}{c} M_{11}=\underset{x}{\sum }\underset{y}{\sum }y^{2}I\left(x^{2},y\right) \end{array}$$

Therefore, the steps of the modified Camshaft algorithm are: first, initialize the filter and calculate the initial center and window of the feature region, second, Kalman predicts the target position, then the target position information is obtained by the Camshaft algorithm and the filter is updated, and finally the updated filter is used to predict the target position in the next frame to achieve continuous tracking of the target. In this paper, we use the Ad boost face detection algorithm to detect the face area of students and send the face detection position to the improved Camshaft algorithm for the calculation to achieve the tracking and positioning of students' faces during study.

The loss function separated when detecting the feature points of internal and external contours, which can lead to an imbalance in locating each key point due to the difference in background and local texture information. In the detection of external contour detection, some interference information may be provided due to the different background information. And in the detection of internal contours, the location information and difficulty of each key point vary. This will lead to an imbalance between the inner and outer contours in training, so separate loss functions need to be computed for the two subsystems to prevent overfitting.

The article "Analysis of Students' Role Perceptions and their Tendencies in Classroom Education Based on Visual Inspection" was retracted in 2024. Reasons: signs of a paper mill; suspected computer-generated content; unreliable results or conclusions; lack of ethics approval or compliance.

The network has three convolutional layers connected with three pooling layers, and the input image pairs have multiple convolutional kernels corresponding to each convolutional layer and output convolutional results. Let the input *t* − *th* convolutional layer be It, which is calculated according to equation (6): where *F*_*x*,*y*,*k*,*x*,*z*_^*t*^ is the input convolutional layer, *F* and *B* are adjustable parameters, and both hyperbolic tangent function and absolute value function are applied to ensure the nonlinearity of the network.

(6) $$\begin{array}{c} C_{i,j,k}^{t}=\left|\tanh\left(\overset{h-1}{\underset{x=1}{\sum }}\overset{h-1}{\underset{y=1}{\sum }}\overset{h-1}{\underset{z=1}{\sum }}I_{i-x,j-y}^{t-1}\cdot F_{x,y,k,x,z}^{t}-B_{k}\right)\right| \end{array}$$

The network model first predicts the boundary region of the face, divides the face into two regional parts, the inner region of the face and the outer region of the face, and then locates the inner and outer feature points of the face and pinpoints the inner feature points, respectively [15]. The external region of the face is divided to facilitate the accurate prediction of the external feature points in the next step, and the divided region can accurately contain all the feature points in the external region of the face, and the boundary of the divided region is expanded by 15% to include as much information as possible to ensure that the divided region contains the possible information of the face. The CNN parameters are shown in Table 1.

Ecological teaching requires teachers to pay close attention to students' emotions and create a harmonious teaching atmosphere, so teachers should be the creators in the teaching environment, creating a good class culture, making class conventions, establishing a good teacher-student relationship and student-student relationship, to establish a good class atmosphere; at the same time, the Internet era requires teachers to have information literacy, sifting valuable information in the complex ocean of information. The Internet era also requires teachers to be information literate, to sift through the complex sea of information, to be discriminators and integrators of information [16]. Therefore, when teachers face the teaching environment, they must be the discriminator and manager of the teaching environment to prevent bad information from entering the classroom and to create a safe environment for students' learning.

The video streams of faces with different periods, various expressions, and a little occlusion were captured by our camera, and then a face feature classifier was used to analyze the video streams, capture, and intercept the face areas in the video streams, and then save the obtained images to a local folder.

The article "Analysis of Students' Role Perceptions and their Tendencies in Classroom Education Based on Visual Inspection" was retracted in 2024. Reasons: signs of a paper mill; suspected computer-generated content; unreliable results or conclusions; lack of ethics approval or compliance.

The images of all testers' faces intercepted with the classifier to capture the eye region and the mouth region as the training set for the eye fatigue judgment network and the mouth fatigue judgment network to carry out the training process of the network model. The dataset for fatigue judgment does not use the student's name as the classification criterion, but the opening and closing of the eyes and the opening and closing of the mouth as the classification labels. Therefore, the data set source for the experiments in this chapter needs to be modified based on the database to provide data for the subsequent training of the network, as shown in Figure 2.

After a long period of study and observation, as well as interaction with students in the class to understand students' daily learning emotions, we can find that when students are more interested in the teaching content and willing to listen to the teacher's lecture, students will participate more in the teaching activities and actively interact with the teacher to answer the teacher's questions, at this time the students' learning state is focused; when students do not understand the content of the teacher's lecture. In this way, multiple corresponding weak classifiers can be directly obtained after multiple cycles, and a strong classifier can be obtained by accumulating and combining these weak classifiers according to the proportion of relative sample weights. When students do not understand the content of the teacher's lecture, their learning state is puzzled; when the teacher's lecture is beyond students' knowledge, their learning state is fatigued; when students feel easy to learn or question the content of the teacher's lecture, their learning state is bored. Therefore, this paper combines literature and actual teaching research to identify four common emotions of students in the learning process as concentration, doubt, fatigue, and boredom, and defines the corresponding facial features of students, such as the corners of the mouth rising and drooping, the eyebrows stretching and frowning, and the eyes closing, respectively.

### 3.2. Experimental Design of Students' Role Perceptions and Tendencies in Classroom Education

To promote the development of education modernization, make up for the shortcomings of current traditional education methods, and help teachers better improve teaching quality, this paper proposes a method for evaluating students' classroom attention that combines head posture and students' emotional changes. This research method can assist teachers to understand students' learning status and emotional changes in the classroom learning process promptly and realize the monitoring and research of students' learning status in the teaching process [17]. While focusing on all students, it is also able to do attention studies on individual students. At the same time, the system reduces the pressure and workload of students and teachers and provides help for teachers to develop and improve their teaching skills. For students, it enables them to receive adequate guidance from their teachers and promotes their learning and physical and mental health development. In the detection of outer contour, some interference information may be provided due to different background information. In the detection of internal contours, the location information and difficulty of each key point are also different. This research method has high practical value for improving the quality evaluation of classroom teaching and is a practical process evaluation method in classroom teaching quality evaluation.

The article "Analysis of Students' Role Perceptions and their Tendencies in Classroom Education Based on Visual Inspection" was retracted in 2024. Reasons: signs of a paper mill; suspected computer-generated content; unreliable results or conclusions; lack of ethics approval or compliance.

The module design and working fundamentals of the student classroom attention evaluation and testing system are mainly: the system collects the students' classroom learning situation. Unlike the one-to-one classroom teaching in the online teaching environment, traditional classroom teaching conducted in a one-to-many manner. The system first needs to track and locate the students' faces for face detection, and then face feature extraction to achieve detection of students' head posture and emotional expression.

Therefore, choosing a good camera is a very important part of the student attention evaluation environment, and is an important hardware resource for the system to obtain data sources on student learning behavior. In the classroom teaching process, students' learning state will present different postures and expressions, and the video images monitored by the camera should be able to cope with the characteristics of complex scenes and polymorphic targets [18]. Therefore, a high-definition camera that can support large-scene recording should be selected, and the panoramic acquisition of the classroom environment ensures the clarity of the classroom teaching environment.

Image pyramid operation not only changes the size of the image but also changes the coordinate labels of the image, so the labels also need to be adjusted accordingly. In this paper, the training data of all training sets are unified and normalized in the process of generating data labels.

The specific way is to calculate the coordinate offset and then label the original image, the normalization method is the same for positive sample, negative sample, and partial sample, the upper left corner of the face frame in the original image is set as (*x*_1_, *y*_*i*_), the lower right corner is set as (*x*_2_, *y*_*z*_), the upper left corner of the face frame in the pyramid transformed image is set as (*x*_3_, *y*) and the lower right corner is set as (*x*_4_, *y*_4_), the specific position relationship is shown in Figure 3 below.

The article "Analysis of Students' Role Perceptions and their Tendencies in Classroom Education Based on Visual Inspection" was retracted in 2024. Reasons: signs of a paper mill; suspected computer-generated content; unreliable results or conclusions; lack of ethics approval or compliance.

The model optimizer in this paper chooses a model based on the adaptive moment estimation method of small batch gradient descent can effectively reduce the fluctuation of parameter updates and eventually get better results and more stable convergence, but it cannot update the learning rate and may jump over the optimal solution in training; Adam is similar to momentum, which can calculate the adaptive learning rate of each parameter, not only the previous squared gradient of decay values but also maintains the previous gradient exponential decay values. Compared with other adaptive learning rate algorithms, Adam converges faster and solves the problems of MGD, which brings about the inability to update the learning rate and slow convergence speed, and ensures the stability of the network while improving the learning effect [19].

The student face area detected and face features extracted, and student attention is analyzed by combining head posture and students' emotional state to make a comprehensive evaluation of students' attention in class. The results of the student attention evaluation are saved to provide data support for teachers to further analyze the teaching research in class, as shown in Figure 4.

Based on this, this paper adopts Base encoding, which is a representation method based on 64 printable characters to represent binary data, although the length of character content will increase after encoding, the dynamic image display in the webpage Base has good results, which can ensure the integrity and stability of the transmission of such non-printable characters in the video, and the distortion of Base is small. The webpage can also display Base synchronously so that students can see their classroom status.

Capture student learning behavior data and ensure the clarity of the image, while saving the high-definition information. The use of fixed large-scene cameras to record the classroom in full clarity can effectively avoid the obscuration of the target [20]. The camera features multiple auto-zooms and auto-iris for clear capture of details in the classroom environment images. At the same time, with the increase in the utilization rate of teaching equipment and mobile terminals, the problem of excessive use of mobile devices by students has also affected the teaching order. Therefore, it is also the responsibility of teachers to effectively manage the use of teaching equipment. The camera can collect students' learning behavior data in class and analyze students' learning status by going to the background. The face detection and tracking algorithm locates students' position in the classroom environment and facilitates teachers to analyze students' classroom attention.

The article "Analysis of Students' Role Perceptions and their Tendencies in Classroom Education Based on Visual Inspection" was retracted in 2024. Reasons: signs of a paper mill; suspected computer-generated content; unreliable results or conclusions; lack of ethics approval or compliance.

## 4. Results Analysis

### 4.1. Performance Results of the Visual Detection Tendency Analysis Algorithm

In this paper, the sliding window model is used to partition the feature sequence into feature subsequence segments. The length of the feature sequence segments is also called the length of the examples, and the length of the examples is also equal to the window size of the sliding window when the examples are partitioned.

In the experiments, using the relative change feature extraction approach of this paper, feature set 3 is selected as the features used for evaluation, and examples of different lengths are divided using sliding windows of different lengths, and the example lengths obtained are 10, 40, 70, 100, 130, 160, and 190.  Figure 5 shows the performance of the two methods with different example lengths. This research method has high practical value for improving the quality evaluation of classroom teaching, and is a practical process evaluation method in the quality evaluation of classroom teaching. From the Figure 5, both methods obtain the same best results (MSE of 0.075) on the validation set. The LSTM-based MIL framework obtains the best results at sequence lengths of 40 and 130, and the method MILDEN in this paper obtains the best results at sequence lengths of 130 and 190, as shown in Figure 5.

As can be seen in the test results, the Faster RCNN using the backbone network is ResNet50 for human figure detection, which has a high accuracy rate but takes too long to meet the real-time requirements of the intelligent classroom vision detection system. While using SSD for human figure detection, the time consuming can barely meet the real-time requirement, but the accuracy is slightly lower, and then adding Gaussian mixture model algorithm, the screen will have a lagging phenomenon. The model distillation method is used to achieve model acceleration, which can meet the real-time requirements and the accuracy rate can also meet the system requirements and get better results.

The unit time is set as t seconds, and the set of open-eye images and closed-eye images of a certain experiment in t seconds is obtained. Not only the previous decay value of the squared gradient is saved, but also the previous exponential decay value of the gradient. Compared with other adaptive learning rate algorithms, Adam has a faster convergence speed, and solves the problem that the learning rate cannot be updated and the convergence speed is slow caused by MGD, which improves the learning effect and ensures the stability of the network. In the image video sequence, the relationship between frame images and time is relative. h is the frame image when the eyes are closed, and H is the total image, where *H* = 15∗*t*, and the relationship between their two ratios can be calculated directly by the formula. According to the mouth area network model, the ratio of the frames with tensor *α* > 1.0 to the total images H per unit time is calculated, and whether there are 50 consecutive frames with tensor >1.0, and the fatigue information and judgment indexes related to the eyes and mouth are combined to make a final judgment on whether the students appear fatigued in the classroom.

The article "Analysis of Students' Role Perceptions and their Tendencies in Classroom Education Based on Visual Inspection" was retracted in 2024. Reasons: signs of a paper mill; suspected computer-generated content; unreliable results or conclusions; lack of ethics approval or compliance.

The threshold values of P were set to 0.2, 0.3, 0.4, and 0.5 for groups 1 to 9. An arbitrary 20-second video (total 300 frames) collected, and the horizontal coordinate is the number of groups with weights, and so on; the vertical coordinate is the accuracy rate, and P with different thresholds are represented by different curves, and the experiment was conducted to determine the optimal group, and the experimental results are shown in Figure 6.

In each experiment, three data were measured, namely, the proportion of closed-eye images to the total number of frames per unit time of the eye denoted as *f*1, the proportion of frames with mouth opening >1.0 to the total number of frames per unit time, denoted as *f*2, and whether there were 50 consecutive frames with mouth opening >1.0, denoted as T. If there were 50 consecutive frames, *T* was denoted as Based on the results of these three experiments, the results of P were calculated and compared to a threshold value of 0.300 to determine whether the state of fatigue was reached. The resulting example lengths are 10, 40, 70, 100, 130, 160, and 190.

The ratio *f*1 of the total number of frames per unit time when the eyes are closed, the ratio *f*2 of the total number of frames per unit time when the mouth opening is greater than 1.0, and whether the mouth opening is greater than 1.0 for 50 consecutive frames and the actual fatigue are determined by the fatigue detection method. To ensure the reliability of the comparison, a large amount of literature in fatigue detection-related fields was read before the comparison, and the overall level of current fatigue detection and mainstream methods were understood, based on which the comparison was made with the method in this paper. The experimental results are compared with the current mainstream PARCLOS judgment method and the emerging PARCLOS-based network model method from four perspectives, such as training time, memory consumption, real-time, and detection accuracy.

The article "Analysis of Students' Role Perceptions and their Tendencies in Classroom Education Based on Visual Inspection" was retracted in 2024. Reasons: signs of a paper mill; suspected computer-generated content; unreliable results or conclusions; lack of ethics approval or compliance.

Finally, the three judgment methods are compared in terms of the accuracy of fatigue detection. According to the current research results, the accuracy of PARCLOS-based deep learning models is generally 90% to 95%, but when the experimenter's face is obscured, this accuracy rate will have a slight decline and is generally lower than 90%. The accuracy of traditional PARCLOS is more affected by various influences and is generally at 75% to 85% when occlusion occurs.

### 4.2. Experimental Results on Role Perception and Tendency

To verify the accuracy of the student classroom attention evaluation detection system in this paper, the actual statistics of students' learning attention at each period were obtained by using the structured observation method on the playback of students' classroom learning videos, and analyzing the students' attention level, participation level and doubt level at each time point. If there are 50 consecutive frames, T is recorded as 0.1, if there are no consecutive 50 frames, T is recorded as 0.0. According to the results of these three experiments, the results of P are calculated and compared with the threshold value of 0.300 to judge whether to enter the fatigue state. The actual statistical results were compared with the system test results to verify the accuracy of the system evaluation. In this paper, students' learning in 30 minutes was selected as a comparison, students' learning was recorded every two minutes, and finally, the difference between the attention evaluation detection system and the actual teaching effect was compared and analyzed. The experimental analysis showed that students' attention was mostly focused on the initial stage of the course, and their learning status would gradually decline as time went by.

After the lesson, we conducted in-depth communication with teachers and students in the form of interviews to analyze the accuracy of the student classroom attention evaluation and testing system. Through interviews with students, it was found that students who watched the video playback after class thought that the evaluation results of the student classroom attention evaluation and testing system were highly accurate following their learning status at that time. Finally, teachers and students agreed that the student classroom attention evaluation detection system is easy to operate and use with high accuracy, which is a good facilitator for classroom teaching, as shown in Figure 7.

The article "Analysis of Students' Role Perceptions and their Tendencies in Classroom Education Based on Visual Inspection" was retracted in 2024. Reasons: signs of a paper mill; suspected computer-generated content; unreliable results or conclusions; lack of ethics approval or compliance.

It further proved that the student classroom attention evaluation detection method can effectively detect students' classroom learning behaviors and is a good process evaluation method that will prompt teachers to fully grasp the classroom teaching content and students' learning, and realize a better application value for classroom teaching while helping teachers to improve teaching quality.

The outgoing, enthusiastic, responsible, independent, and caring personality traits of student leaders are more evident, and they are constantly being honed and their personalities are changing as they deal with conflicts between teachers and students and between students and teachers in the context of more complex interpersonal relationships. The recognition results have higher accuracy and better application value. Through interviews with students, it was learned that the students watched the video playback after class and believed that the evaluation results of the students' classroom attention evaluation and detection system were in line with the current learning state and had high accuracy. Individuals with higher psychological resilience tend to treat life's unsatisfactory changes as special tests, and they are optimistic about such changes. Optimism is an individual's positive cognitive evaluation, not only in the face of sudden change situations, but they also show a positive expectation when faced with the teacher role, as shown in Figure 8.

Through the experimental results of fatigue detection above, it can be found that the traditional single judgment index PARCLOS is problematic in judgment. For example, the 4 videos, with more eyes closed in contemplation, is characterized by the fact that although the proportion of eyes in the closed state is larger, it cannot be judged singularly as having entered fatigue because its mouth does not show the performance in the related fatigue state. In addition, the fifth video characterized by a lower proportion of frames with eyes closed, but the frequency of yawning was obviously higher, and the mouth opened and closed widely for 50 consecutive frames, so it could judge to be fatigued. In this experiment, a total of 50 video streams to be tested were input, each of which was 20 seconds, either in fatigue or in normal, and 46 videos were judged correctly, with an accuracy rate of 92%, achieving the expected goal of the experiment.

## 5. Conclusion

This paper designs and implements a student concentration detection model system based on online educational video content based on the self-recorded database and the existing database as the database, and the system collects student classroom video data through the client and transmits it to the server, and the server realizes the classroom status judgment of students by calling two modules of face detection and fatigue detection and returns the output results to the client for feedback. Therefore, it can be judged that it belongs to the fatigue state. In this experiment, a total of 50 video streams to be tested were input, each of 20 seconds, either in fatigue or normal, 46 videos were judged correctly, the accuracy rate was 92%, and the expected goal of the experiment was achieved. The face detection module is responsible for recognizing whether there is a human face in the video, eliminating excess noise interference, and locating the detected face feature points, while the fatigue detection module is responsible for recognizing the changes in students' eyes and mouths, determining whether students are fatigued, and then analyzing the students' concentration level. The system is tested and evaluated to understand the accuracy and real-time performance of the analysis system, and then two strategies are proposed to improve the real-time performance and accuracy of the system. In this paper, the cascaded convolutional neural network is used to accurately locate the facial feature points of the face, which provides a strong guarantee for the estimation of students' head posture. Four student classroom emotional features are proposed based on the emotional changes of students' classroom learning, and the comprehensive evaluation and analysis of students' attention are realized by combining the changes of students' head posture and facial expression features. The experimental results and analysis show that the system has good accuracy and stability, and at the same time can effectively analyze students' attention in a classroom environment, which provides a research direction for the modernization of education and more software into the classroom environment.

The article "Analysis of Students' Role Perceptions and their Tendencies in Classroom Education Based on Visual Inspection" was retracted in 2024. Reasons: signs of a paper mill; suspected computer-generated content; unreliable results or conclusions; lack of ethics approval or compliance.

## Figures and Tables

**Figure 1:** Visual detection principal framework.

**Figure 2:** Relationship between basic emotion and expression tendency features.

**Figure 3:** Label normalization of the boundaries of the character recognition box.

**Figure 4:** Partial eye network model classification.

**Figure 5:** Comparison of accuracy test results of different human figure detection algorithms.

**Figure 6:** Effect of some parameters on the accuracy of the experiment.

**Figure 7:** Comparison of Doubt Levels.

**Figure 8:** Experimental results.

**Table 1:** Configuration of face external contour parameters.

The internet	Input	Convolution kernel and stride	Output
Convolution 1	60 × 60 × 64	5 × 5/1	30 × 60 × 3
Pooling 1	56 × 28 × 64	2 × 2/2	56 × 28 × 64
Convolution 2	28 × 28 × 64	5 × 5/1	28 × 14 × 64
Pooling 2	24 × 12 × 96	2 × 2/3	12 × 24 × 48
Convolution 3	12 × 12 × 96	4 × 4/1	12 × 12 × 96
Pooling 3	10 × 5 × 128	2 × 2/2	10 × 5 × 128
Local connection layer	5 × 5 × 128	3 × 3/1	5 × 5 × 128

## Data Availability

The data used to support the findings of this study are available from the corresponding author upon request.

## References

[1] Birgili B., Seggie F. N., Oğuz E. (2021). The trends and outcomes of flipped learning research between 2012 and 2018: a descriptive content analysis. *Journal of Computers in Education*.

[2] Berman N. (2020). A critical examination of informal learning spaces. *Higher Education Research & Development*.

[3] Ozkal N. (2019). Relationships between self-efficacy beliefs, engagement and academic performance in math lessons. *Kıbrıslı Eğitim Bilimleri Dergisi*.

[4] Toropova A., Myrberg E., Johansson S. (2021). Teacher job satisfaction: the importance of school working conditions and teacher characteristics. *Educational Review*.

[5] Schipper T. M., de Vries S., Goei S. L., van Veen K. (2020). Promoting a professional school culture through lesson study? An examination of school culture, school conditions, and teacher self-efficacy. *Professional Development in Education*.

[6] Svalberg A. M. L. (2018). Researching language engagement; current trends and future directions. *Language Awareness*.

[7] Lockman A. S., Schirmer B. R. (2020). Online instruction in higher education: promising, research-based, and evidence-based practices. *Journal of Education and e-Learning Research*.

[8] Hidayati N. A., Waluyo H. J., Winarni R. (2020). Exploring the implementation of local wisdom-based character education among Indonesian higher education students. *International Journal of Instruction*.

[9] Song P., Wang X. (2020). A bibliometric analysis of worldwide educational artificial intelligence research development in recent twenty years. *Asia Pacific Education Review*.

[10] Carpenter S. K., Witherby A. E., Tauber S. K. (2020). On students’(mis) judgments of learning and teaching effectiveness. *Journal of Applied Research in Memory and Cognition*.

[11] Yates A., Starkey L., Egerton B., Flueggen F. (2021). High school students’ experience of online learning during Covid-19: the influence of technology and pedagogy. *Technology, Pedagogy and Education*.

[12] Allen K. A., Kern M. L., Vella-Brodrick D., Waters L. (2018). Understanding the priorities of Australian secondary schools through an analysis of their mission and vision statements. *Educational Administration Quarterly*.

[13] Bouilheres F., Le L. T. V. H., McDonald S., Nkhoma C., Jandug-Montera L. (2020). Defining student learning experience through blended learning. *Education and Information Technologies*.

The article "Analysis of Students' Role Perceptions and their Tendencies in Classroom Education Based on Visual Inspection" was retracted in 2024. Reasons: signs of a paper mill; suspected computer-generated content; unreliable results or conclusions; lack of ethics approval or compliance.

[14] Asino T. I., Pulay A. (2019). Student perceptions on the role of the classroom environment on computer supported collaborative learning. *Tech Trends*.

[15] Kumar J. A., Bervell B., Osman S. (2020). Google classroom: insights from Malaysian higher education students’ and instructors’ experiences. *Education and Information Technologies*.

[16] Bevilacqua D., Davidesco I., Wan L. (2019). Brain-to-brain synchrony and learning outcomes vary by student–teacher dynamics: evidence from a real-world classroom electroencephalography study. *Journal of Cognitive Neuroscience*.

[17] Lancaster J. R., Lundberg C. A. (2019). The influence of classroom engagement on community college student learning: a quantitative analysis of effective faculty practices. *Community College Review*.

[18] Koç Ö., Altun E., Yüksel H. G. (2022). Writing an expository text using augmented reality: students’ performance and perceptions. *Education and Information Technologies*.

[19] Pánek J. (2019). Emotional maps: participatory crowdsourcing of citizens perceptions of their urban environment. *Cartographic Perspectives*.

[20] Vermote B., Aelterman N., Beyers W., Aper L., Buysschaert F., Vansteenkiste M. (2020). The role of teachers’ motivation and mindsets in predicting a (de) motivating teaching style in higher education: a circumplex approach. *Motivation and Emotion*.

